This article has been retracted.

# Revamping of Chronic Respiratory Diseases in Low- and Middle-Income Countries

**DOI:** 10.3389/fpubh.2021.757089

**Published:** 2022-02-21

**Authors:** Ling-Hui Zeng, Musaddique Hussain, Shahzada Khurram Syed, Malik Saadullah, Qurratulain Jamil, Ali M. Alqahtani, Taha Alqahtani, Nadia Akram, Imran Ahmad Khan, Sajida Parveen, Tehreem Fayyaz, Mobeen Fatima, Saira Shaukat, Najia Shabbir, Mehwish Fatima, Aisha Kanwal, Muhammad Qasim Barkat, Ximei Wu

**Affiliations:** ^1^Department of Pharmacology, Zhejiang University City College, Hangzhou, China; ^2^Department of Pharmacology, Faculty of Pharmacy, The Islamia University of Bahawalpur, Bahawalpur, Pakistan; ^3^Department of Basic Medical Sciences, School of Health Sciences, University of Management and Technology Lahore, Lahore, Pakistan; ^4^Department of Pharmaceutical Chemistry, Government College University, Faisalabad, Pakistan; ^5^Department of Pharmacy Practice, Faculty of Pharmacy, The Islamia University of Bahawalpur, Bahawalpur, Pakistan; ^6^Department of Pharmacology, College of Pharmacy, King Khalid University, Abha, Saudi Arabia

**Keywords:** asthma, COPD, tuberculosis, bronchiectasis, emphysema–pneumonia–bronchiolitis–smoking–fibrosis–histiocytosis

## Abstract

Low- and middle-income countries (LMICs) endure an asymmetrically high burden of worldwide disease and death caused by chronic respiratory diseases (CRDs), i.e., asthma, emphysema, bronchiectasis, and post-tuberculosis lung disease (PTLD). CRDs are firmly related with indigence, infectious diseases, and other non-communicable diseases (NCDs) and add to complex multi-disease with great impact on the lives and livelihood of those affected. The pertinence of CRDs to health and demographic wellbeing is relied upon to increment in the long time ahead, as expectations of life rise and the contending dangers of right on time youth mortality and irresistible infections level. The WHO has distinguished the counteraction and control of NCDs as an earnest improvement issue and crucial for the sustainable development goals (SDSs) by 2030. In this review, we center on CRDs in LMICs. We examine the early life roots of CRDs, challenges in their avoidance, identification and administration in LMICs, and the pathways to resolve for accomplish valid widespread wellbeing inclusion.

## Introduction

Non-communicable diseases (NCDs) are a vital root of morbidity and mortality. In low- and middle-income countries (LMICs) (1), round about 70% of worldwide deaths are reported from NCDs with an elevated threat of dying (2). The purpose of the Sustainable Development Goals (SDGs) of the United Nations is to overcome the threat of precocious fatalities from NCDs by a third by 2030 (3). The ordinary and relatively ignored NCDs that twain the life cycle are chronic respiratory diseases (CRDs), such as asthma, chronic obstructive pulmonary disease (COPD), bronchiectasis, and post-tuberculosis lung disease (PTLD). They are often related with the high level of patient and healthcare prices, morbidity, and threat of mortality by reason of constant manifestation; activity, limitations, and Irregular aggravation need intense care. They inadequately influence poor people in all countries, but mainly in LMICs where assets for research, prevention, and management are rare (4). The recent Lancet Commission on injuries has helped to raise the issues of justice and probity for the poor people of the whole world (5). This evaluation fixates on continual breathing ailment in LMICs. Even though, dearth and social destitution are worldwide matters, we accept that. People who lived in LMICs encountered a specifically hard coalition of destroying early life and environmental exhibition, tasking social and political interpretation, and poor access to prime trait health facilities. We talk about the formative years of CRDs in LMICs and possible strategies to the obstruction of the disease. We propose tactics for research and clinical capacity reinforcement, for both the prevention and management of CRDs. We propose tactics for research and clinical capacity reinforcement, for both the obstruction and regulation of CRDs, and suggest pathways to a solution that would impart to attain international tasks for health including to overcome morbidity and inopportune mortality and attaining worldwide health coverage.

## Early Life Origins of CRD

Evidence that has mainly been received in high-income countries (HICs) shows that the *in-utero*, infant, child, adults, and surrounding conditions are extremely important for lung development, with preschool lung function, and early adult lung functions, into at least the seventh decade of life (6, 7). Even though, related data from LMICs are rare, the same association probably holds true in these countries (8). Common to both settings are detrimental *in-utero* and early childhood exposures. These can disturb lung development such that individuals fail to reach an optimal peak in early adulthood, with increased CRDs later in life. In LMICs, the increased pervasion and severity of many of these harmful early life exposures might explain the lower lung volumes observed in asymptomatic non-smoking age- and height-matched adults in HICs and in many sub-Saharan African settings (9). Epidemiological evidence is provided to show the association of prenatal or perinatal exposure to air pollutants with various adverse birth outcomes, such as preterm birth, lower birth weight, and lung developmental defects. Interventions to mitigate early life exposures might be crucial for the prevention of CRDs in LMICs (7, 10–12), because of the potential value of *in-utero* and adult lung function and early childhood exposures, the high incidence of these negative effects on one's wellbeing, and the fact that they are so common. In early life exposures and treatments in LMICs, the importance of exposures in the prevention of CRDs may be critical in the least developed countries.

### *In-utero* Exposures

Tobacco smoking changes lung structure and function and affects the immune system of fetus (6). A health study in South Africa—one of first births cohorts in Sub-Saharan Africa-reports, infants of third mothers who smoked during pregnancy had lower tidal volume and higher lung clearance indices at age 6 weeks than infants of non-smoking women (13, 14). Depression, prenatal stress, bad living conditions and intimate partner, and neighborhood violence are issues faced by women around the world. Maternal stress and depression are negatively connected with measures of neonatal health and positively connected with respiratory morbidity in children (15, 16). Maternal alcohol exposure during pregnancy negatively affects lung function at 6 weeks. This effect disappears by 1 year (8, 13). The number of HIV in women of childbearing age is high in many LMICs. The introduction of test and treat approaches to combination antiretroviral treatment (cART) and dedicated programs to prevent mother-based-to-child transmission have decreased rates of perinatal infection (17). Preterm birth is related to increased breathing and lung-related signs of sickness. Premature births occur in 10% of all live births around the world, 80% of these are in LMICs (18, 19).

### Childhood Exposures

Maternal smoking and environmental tobacco smoke (ETS) exposure influence infant lung development and are associated with childhood upper and lower respiratory tract infection, wheezing, or asthma (20). Bacterial and viral infections are common in LMICs in early childhood. Some of the most common viral pathogens respiratory syncytial virus, rhinovirus, adenovirus, and influenza A are detected in children with acute lower respiratory tract infections in LMICs (21). A common and serious illness, which affects children of all age groups, is community-acquired pneumonia (22). In LMICs, infectious, maternal, neonatal, and nutritional diseases are still major contributors to disease burden. By contrast, in upper middle income and HICs, NCDs are predominate (23). In LMICs, pneumonia is the major root of mortality in children with an estimated incidence of 0.2–0.3 episodes per-child year (24). In Sub-Saharan Africa, lower respiratory infection in early childhood is an independent risk factor for reduced lung function by 1 year of age; however, pneumococcal vaccine is still only available to ~50% of children around the world, despite its introduction two decades ago (13, 25).

#### Tuberculosis in the Lungs

Children under the age of 15 account for 11% of new cases of tuberculosis worldwide (26), and pediatricians with LMICs regularly record a high burden of post-tuberculosis squeal, such as bronchiectasis and lung destruction, in children who successfully complete care (27).

#### HIV Infection That Lasts a Long Time

In LMICs, a large number of children who were initially born with vertically transmitted HIV are now approaching adulthood (28). These long-term survivors have a high prevalence of CRDs, such as bronchiectasis, obliterans bronchiolitis, and reduced lung function (27, 28). Deficits are more serious in people who have been diagnosed late and started antiretroviral treatment late (29).

#### Dietary Advice

Maternal and childhood malnutrition are becoming more common in LMICs (30), resulting in fetal growth problems. Restriction, stunting, waste, and food isolation are also examples of nutrient isolation. Not only children with deficiencies, but also those who are overweight or obese (31, 32) based on the limited information available. It seems that *in-utero* early childhood, hunger has a negative impact on lung formation that continues into adulthood adolescence. Obesity has also been linked to long-term airway disease in LMICs, it is been linked to asthma and in HICs (33).

#### Pollution of the Air

Indoor and outdoor air exposures can have an effect on a child's lung health. The connection between the two early childhood biomass fuel exposure and lung development is unknown. Delayed penetration of clean burning stoves into Guatemalan households (child age 18–57 vs. <6 months) was linked to lower lung growth rates (34). Results from a clean stoves intervention sample in rural Malawi revealed a minor but statistically important gap (0.2 Z scores) in the forced vital capacity (FVC) of children from households who had previously received a clean burning stove (35). In HICs, increases in outdoor air emissions over time have been linked with improved lung function (36). There has been a connection between diesel exposure and bad asthma results, and this may be especially true for children. Significant in LMICs, where trucks are often in poor condition maintained, unrestricted petrol, and driving in close quarter's proximity of human settlement (37–39).

#### Direction of Solutions

In order to prevent CRDs in LMICs, attention must be paid to prenatal and early childhood exposures, which influence the development of the disease. The evolution and health of the lungs over the course of a person's life, many of these exposures can be regulated for public health reasons. Interventions and poverty among mothers are at the root of the problem. Maternal care programs must be reinforced to preserve the physical and mental health of women of childbearing age and mothers, enhance access to high-quality prenatal care, and enhance maternal education on children's nutrition and immunization. Programs that assist HIV-positive mothers in preventing perinatal transmission and providing early HIV testing for their children must be continued. We recommend that early child health programs should be enhanced, with safe access to high-quality nutrition and effective vaccination. Given the anticipated negative consequences of air pollution on lung development, we recommend that endeavor to enhance changes in cooking and ventilation techniques should be continued as a potentially low-cost plan for improving child health (40). Political interventions, such as taxes and successful advertisement regulation legislation, would be necessary to reduce smoking exposure; it will most likely be necessary for cigarettes, nicotine, and indoor and outdoor air pollution (41). Such efforts could be particularly useful due to increased marketing and intervention. LMICs are becoming more vulnerable with public health efforts by tobacco, alcohol, food, inadequate national regulatory mechanisms (4), and soda industries. Many of these healthcare system and policy changes are large in nature and have the potential to help people with diseases other than CRDs. However, without them, the considerable burden of CRDs in LMICs is likely to persist.

## Chronic Obstructive Pulmonary Disease

Chronic obstructive pulmonary disease afflicted 212.33 million adults worldwide in 2019, according to the global burden of disease figures (42). Primary record on the worldwide burden of ailment shows significant variability in the prevalence, reasons, scientific presentation, and mortality among and inside LMICs (43). These discrepancies are mostly due to a lack of spirometry and epidemiological evidence, but they are exacerbated by disagreements about the concept of COPD. For example, it is unknown if fixed percentages, percent expected cutoffs, or lower limit of natural boundaries should be used to distinguish irregular outcomes, what reference ranges should be used for estimation standardization, and whether all patients with fixed airflow obstruction should be considered COPD (9). Despite this problem, community-based evidence shows that airway obstruction is common in Latin America, between 6 and 20% of people are obstructed (44–46). In Sub-Saharan Africa, the rate is 5–24% (47–50). LMICs are thought to be responsible for 71% of global COPD strain, 84% of global COPD deaths, and 84% of global COPD disability-adjusted life year (DALY) around the world (42). Even though, tobacco smoking is still a significant risk factor for airway blockage in LMICs, between a third and a fifth of instances occur in persons who have never smoked, and a significant fraction of these instances are likely connected to biomass usage for cooking and heating, particularly among women (51–55).

### The Prognosis

In LMICs, high degrees of under-diagnosis and misdiagnosis of COPD are determined (56, 57). Results from recent national COPD surveys show that more than one-third of the world's population suffers from this disease, 80% of COPD cases detected by spirometry go undiagnosed in normal clinical care (58). Individuals with a minor illness and no prior experience with exacerbations or admissions are less likely to result in a positive outcome. Ethnicity, socioeconomic background, and the lack of interaction with healthcare providers have also been identified as a risk factor for under-diagnosis, suggesting that broader socioeconomic determinants are also important (56–58). As previously mentioned, inadequate worldwide access to spirometry for diagnosis is likely a major stumbling block.

### Management

Non-pharmacological therapies are often used in the treatment of smoking-related COPD (supported smoking abstinence, pneumococcal and influenza vaccination, and pulmonary rehabilitation). In addition to pharmacological treatment with inhaled therapies, short-acting beta agonist (SABAs), long-acting beta agonists (LABAs), and short-acting and long-acting muscarinic antagonists, inhaled corticosteroids (ICs) according to the severity of the disease. In LMICs, these measures are underutilized. A population-based survey in Latin America shows that just half of the smokers received medical advice, according to a new study. A quarter were given some kind of respiratory drug, and access to the influenza vaccine was ineffective (59, 60). According to the Public Use Micro data Area (PUMA) survey results, the most commonly used treatment in primary care was SABA-inhaled treatment, with long-acting bronchodilators (LABA) and ICs being used less frequently (61). There have been no clinical trials to determine the best pharmacotherapy for non-smoking-related COPD, such as disease caused by biomass pollutant peril in LMICs, which could vary from those prescribed for smoking-related COPD.

### Direction of Solution

Better epidemiological evidence, correct diagnosis, and adequate clinical treatment for COPD in LMICs are all instantly needed (62, 63). Increasing consciousness among patients and clinicians, using licensed standardized protocols for diagnosis and treatment, greater access to spirometry, expanded use of inhaled treatments, improved education for both patients and healthcare providers, and better access to long-term follow-up are some of the interventions that could be needed. COPD, on the other hand, is more common in HICs that has been linked to a variety of systemic consequences, such as cardiovascular disorder, malignancy, osteoporosis, stress, and anxiety (64). As a result, it is important to see if the same results are observed in LMICs, because if they are, programs to overcome this multi-morbidity would almost certainly be required. Increasing access to non-pharmacological treatments that are less expensive, such as smoking abstinence and pulmonary therapy, should be prioritized and tailored to unique cultural environment (65). Smoking is also the leading cause of the COPD worldwide and attempts to transfer lessons learned in HICs about public health and policy approaches to control to LMICs, in order to minimize both direct and passive exposure, would take continued long-term help. In both high- and low-income environments, data on the risks, existence, consequences, and treatment of non-smoking associated airway obstruction are required.

## Asthma

Asthma is the most ordinary CRD in the world, influencing 262.4 million people in 2019 (42), with LMICs leading 96% of asthma-related worldwide deaths and 84% of DAIY worldwide. Asthma-related diseases and deaths, on the other hand, are entirely avoidable (66).

### The Prognosis

In LMICs, the Global Initiative for Asthma (GINA) recommends using a syndromic approach to asthma diagnosis. However, it emphasizes the significance of using peak flow control or spirometry with reversibility checking to measure variations in air flow for validation (67). In LMICs, access to these equipment is limited, substantially limiting diagnostic capabilities (68). In LMICs, asthma is usually under-diagnosed in children and adults, and when it is diagnosed, it is generally more severe (69, 70).

### Management

Inhaled corticosteroids are used to treat chronic asthma and improve symptom control and lowering hospital visits and death rates (71). For adolescents and adults in therapy stages 1 and 2, GINA now recommends using inhalers containing ICs and the rapid-onset LABA formoterol as needed (67, 72). Large clinical trials show that this approach is equivalent to or better than using regular ICs with as-needed short-acting 2 agonists (SABAs) for minimizing the threat of acute exacerbations, and that it uses a much lower dose of ICs with no clinically significant difference in symptom control, at least in teenagers and adults over the age of 12 (73–76). Similarly, in moderate-to-extreme asthma, using a mixture of ICs and formoterol for maintenance and reliever treatment decreases severe exacerbations compared to using standard ICs and LABA therapy with a SABA reliever (77). For this reason, if combined ICs and bronchodilator preparations are not available or reasonable for moderate asthma, separate ICs can be used whenever a SABA is taken. Despite these recommendations, ICs are often under-prescribed, inaccessible, or unaffordable to patients and people with asthma in LMICs, who rely on inhaled bronchodilators alone, or take oral bronchodilators Instead, use salbutamol, theophylline, or prednisolone preparations (68, 70, 78, 79). The ability of the healthcare system to provide long-term follow-up and prescription titration for symptom monitoring is limited and patient and clinician awareness of the need for chronic treatment could be inadequate, with 52–76% loss of follow-up seen within 1 year in pilot projects in China, Benin, and Sudan (70, 78, 79).

### Direction of Solutions

Global asthma treatment methods for LMICs may be tailored for national use (67). The implementation will necessitate healthcare workers with advice and training a number of cadres to increase clinical identification of asthma, to encourage the use of syndromic identification, and to ensure that adequate preventer treatment are prescribed appropriately. A major need exists for improved access to diagnostic tools (peak flow meters and spirometry) and training in their use. Similarly, access to affordable quality-assured asthma medicines listed on the WHO A list of essential medicines (panel 1) is needed. Education would be necessary to ensure the safety of both patients and caregivers. The proper use of inhalers, with a focus on the value of ICs and inhaler technique preparation and spacer to improve drug delivery in adults and infants will be needed. Healthcare facilities that can accommodate in LMICs, asthma follow-up is uncommon, but it is critical for avoiding over-reliance on emergency care, maintaining long-term symptom management, and reducing morbidity and mortality.

## Bronchiectasis

In recent years, the confirmed incidence of non-cystic fibrosis bronchiectasis in HICs has increased to 566 per 100,000 (80), with disease prevalence and severity is linked to rising age and female gender (81). While there are few epidemiological statistics on bronchiectasis in LMICs (82), the few data that are available show that the prevalence, reasons, and risk factors for bronchiectasis vary significantly to those in most HICs, with more post-infectious disease, a correlation with HIV infection, a greater burden of acute disease in younger adults, and distinctions in colonizing or infecting microbiology (80, 83, 84).

### The Prognosis

In LMICs, bronchiectasis is difficult to diagnose. The clinical appearance is close to see in people in HIC with persistent cough and sputum production in adults, and children's inability to succeed is often linked with repeated infections and frequent, extreme respiratory symptoms. In several low-resource environments, however, patients with tuberculosis that present with a high tuberculosis rate, these symptoms are mainly managed as tuberculosis suspects who have not been tested for underlying CRDs. The use of CT imaging as the gold standard diagnostic technique for bronchiectasis is highly recommended in international guidelines, but CT imaging is not applicable to the majority of people living in LMICs. There is evidence to justify the use of a simple chest x-ray for the diagnosis of bronchiectasis. Few recommendations advocate the use of a chest x-ray for the investigation in LMICs, with recurrent respiratory problems, in general.

### Management

In HIC, management of bronchiectasis is becoming more individualized and based on addressing so-called treatable traits, with the use of airway clearing tools, vaccination against pneumococcal and influenza, treatment of organisms that are infecting or colonizing, and intercurrent fungal and non-tuberculosis mycobacterial disease needs early detection and active management (85). Individualized treatments are not readily available in LMICs, and no recommendations for the diagnosis and treatment of bronchiectasis in resource-poor settings have yet been established to our knowledge.

### Direction of Solutions

In LMICs, more effective investigation and treatment methods for persistent cough in children and adults are required. Standardized protocols for decentralized treatment are needed, with an emphasis on programmatic interventions that are both practical and scalable (80). These recommendations must provide adequate inspection for active tuberculosis disease in environments with a high tuberculosis burden, but also recognition of underlying CRD when tuberculosis is ruled out. This will necessitate more seamless incorporation of tuberculosis care with other respiratory or surgical services. Healthcare staff is being educated on persistent productive cough is caused by bronchiectasis, to make this possible, usable and inexpensive diagnostic approaches in the absence of CT imaging are needed. In children in South Africa, patient-centered, low-cost tools, such as airway clearing, have been seen to be appropriate and efficient and should be optimized for use in LMICs (86). To advise population-level antibiotic guidelines, a better understanding of the microbiology of bronchiectasis in both children and adults is needed.

## Post-tuberculosis Lung Disease

Survivors of pulmonary tuberculosis, estimated to number 58 million worldwide so far (26), have a 2-to-4-fold chance of having persistently irregular spirometry (airway obstruction and poor FVC patterns) after tuberculosis treatment compared to those who have never had tuberculosis, Bronchitis, parenchymal cavitation and destruction, and fibrotic alteration are all common conditions (87–90). As seen on imaging, there is a lot of diversity in the world. Residual pathology's prevalence, variations, and severity, however, bronchiectasis or pathological spirometry is believed to be the cause, more than a third of tuberculosis patients had pulmonary tuberculosis survivors (90–92). Long-term persistent respiratory complications, repeated respiratory exacerbations, and increased lung function loss are all risks for people with PTLD. Survivors of tuberculosis are at a high risk of recurrence, reactivation, or reinfection of tuberculosis disease (93). Chronic respiratory problems, on the other hand, put them in jeopardy of being subjected to irrational and unjustified tuberculosis retreatment (94), subjecting them to additional drug side effects, stigma, and healthcare costs are also factors to consider (95). Adult tuberculosis (TB) survivors have a nearly 3-fold higher death rate than the general population, however, the link between PTLD and mortality is uncertain (96). Moreover, 1 million of the 10 million yearly occurrences of acute pulmonary TB in the world occur in children (26), but little is known regarding the burden and consequences of PTLD in this group.

### The Prognosis

Spirometry or chest x-ray imaging abnormalities may indicate PTLD, but these procedures are not regularly performed after tuberculosis treatment has been completed and they may not be available at the point-of-care in decentralized TB treatment programs. As a result, the majority of people with residual PTLD are discharged without a diagnosis or a plan for follow-up treatment in LMICs (91). The identification of recurrent TB in people with PTLD can be difficult: nucleic acid amplification tests' sensitivity is lowered in TB survivors, and the effectiveness of screening methods, such as the WHO symptom screen and chest radiography in individuals with PTLD, is unknown (97, 98).

### Management

Existing international and national TB recommendations pay little attention to post-tuberculosis morbidity, and there are no evidence-based guidelines for the diagnosis and therapy of PTLD in LMICs (99, 100). Existing strategies are based on COPD and bronchiectasis treatment models and include cannabis and smoking education, which are prevalent co-exposures in patients with TB. Exercises to clear the airways, vaccines according to national standards, and the use of inhaled bronchodilators for reversible airway blockage are all recommended (101). Because of the elevated risk of chronic mycobacterial disease and other respiratory infections, ICs should not be used (102–104). Rehabilitation of the lungs can aid in the enhancement of one's quality of life (105). Even though sputum culture is the gold standard device for the conclusion of recurrent tuberculosis infection and medicates vulnerability testing in this gather, culture is regularly not accessible in LMICs and is not achievable in young children. More research into the effectiveness of TB screening and diagnostic techniques in pulmonary TB survivors and individuals with PTLD is needed.

### Direction of Solutions

Following the conclusion of TB treatment, pulmonary TB survivors can be screened for persistent lung pathology, with the goal of continuing to monitor and intervene. However, given the limited resources available, more information is needed in LMICs to support choices on how this should be done, which patients might benefit from continued follow-up, and before implementing this strategy, and the efficacy and cost-effectiveness of healthcare treatment for this population. In addition, clear evidence-based recommendations are required for the prognosis and management of those who are not detected at the end of therapy but re-appear with persistent respiratory problems years later. Improved methods to the identification of recurrent TB illness will necessitate the integration of TB and CRD services in order to enhance PTLD diagnosis and management (106). We propose that any packages of post-TB treatment should also address the larger cardiovascular, psychological, and socioeconomic morbidities that tuberculosis survivors experience (107).

## Strengthening of Healthcare Programs

Strong health infrastructure, capable of delivering reliable and responsive care throughout the life cycle would be critical for the prevention and treatment of CRDs and NCDs in LMICs and must include the availability of comprehensive maternity care. The WHO has identified six important building elements that must be addressed in the development of these systems: service delivery, health workforce, health information systems, availability to key drugs and vaccinations, finances, and leadership or governance are all important factors to consider (Figure 1) (108). Numerous key flaws have been recognized in those regions with respect to respiration care in LMICs. The availability of healthcare surveillance data for respiratory diseases other than tuberculosis is limited (109), limiting the potential of countries to recognize and plan for the healthcare needs of their inhabitants. There are no reliable metrics for monitoring and evaluating priority CRD programs. National guidelines for the management of CRDs are also scarce, with just 64% of countries having them according to the seventh NCD national capability study 2019 (110).

**Figure 1:** WHO six building blocks of the health system, together with aims and desirable attributes.

Spirometry and imaging are important diagnostic tools, which are insufficient, in 2019, just 45% of primary care institutions had peak flow or spirometry, compared to 88% for blood glucose testing (111). Preventive interventions, such as the quality of vaccinations, dietary assistance, and smoking abstinence services is inadequate (112). Most importantly, the healthcare workforce is badly equipped to provide respiratory care, with a scarcity of respiratory specialists (113–116), and the majority of care is provided at the primary care level by untrained nurses (117). In the following paragraphs, solutions to some of these challenges are described.

### Integrated Delivery of CRD Care

In LMICs, front-line primary care workers are required to offer preventative and curative treatment to both children and adults for infectious and non-infectious illnesses. As a result, CRD services must be well-integrated into larger services and tailored to local requirements. To this purpose, many integrated care techniques have been developed for use in LMICs (118, 119). The WHO Practical Approach to Lung Disease (PAL), which was designed in part to enhance TB case discovery, was one of the first models to focus only on respiratory disorders. These were followed by tools with a more broader reach, such as the WHO Package of Non-communicable Disease Interventions (PEN) (120). Children, adolescents, and adults can benefit from the WHO's Integrated Management of Adolescent and Adult Illness (IMAI) (121) and Package of Care Kit (PACK) (122). For example, PACK offers a decision-making tool that may be used in a variety of clinical scenarios and is accessible in both print and computer formats (123–126). It incorporates local management principles and evidence, is updated on a regular basis, and is backed up by case-based, interactive training on-site (122, 123). Qualitative results show that this integrated care strategy is successful in enhancing CRD services, such as asthma treatment, TB detection, and appropriate hospital referrals (127–129). We believe that in LMICs, respiratory and TB care should be closely connected. Patients with acute and CRD typically appear with exacerbating respiratory symptoms, and in TB-endemic areas, active TB illness is routinely investigated. However, if these tests come back negative, it is critical to examine other respiratory illnesses. Patients with PTLD after the end of TB therapy would benefit from clear and efficient integrated care pathways, as well. Finally, NCD programs in LMICs should think about incorporating palliative care support in their services. This is especially relevant for CRDs, which are typically incurable, progressive, and can cause painful symptoms like severe dyspnea. This type of incorporation would necessitate cultural understanding, personnel and patient education, the advancement of symptom management strategies, and access to opioid drugs (130).

### Improving Medical Interface Accessibility

The funding of diagnostic instruments, such as spirometry and imaging, and training of clinical personnel on how to perform tests, maintain quality control, and appropriately interpret data are two specific difficulties in obtaining diagnostic technologies at the primary care level (131). Decentralization may be facilitated by advances in the creation of dependable and portable spirometry, ultrasonography, and chest x-ray equipment for community-based diagnosis, but services might be more sustainable if they are supported by education and access to equipment maintenance services (132). More advanced diagnostics, such as CT imaging, complex lung function testing, and bronchoscopy, will almost certainly remain the domain of tertiary centers in LMICs, but these tools are useful in the training and retention of specialists and the development of research capacity, so some investment in their centralized use may be beneficial.

### Enhancing Treatment Accessibility

Inhaled corticosteroids were commonly accessible in 19% of low-income countries in 2019, compared to 96% of HICs, and bronchodilators in 55 and 100%, respectively, despite the fact that numerous important respiratory drugs are on the WHO's list of essential medicines (panel 1). Even when they were accessible, these treatments were typically out of reach for people in LMICs. Despite being among the most cost-effective interventions for CRDs and relevant to the prevention and management of other NCDs, such as cardiovascular disease and cancer, access to non-pharmacological interventions, such as pulmonary rehabilitation and smoking cessation services, is insufficient in LMICs. There are few educational program aimed at improving self-management, promoting health literacy, and combating stigma. Access to these therapies requires immediate advocacy. In LMICs, there are significant data gaps regarding the cost-effectiveness of recently indicated therapies for respiratory disorders, such as ICS–formoterol therapy as needed (and on a frequent basis) in asthma and dual LAMA and LABA treatment in COPD. Rather than presuming unaffordability, the quality pharmacoeconomic analysis should influence plans for broadening the alternatives and tactics offered as necessary medications for respiratory disorders in LMICs. Efforts to adapt and incorporate non-pharmacological therapies into care programs will be necessary and strategies to ease the economical delivery of quality-controlled supplies of these drugs (133). Improving access begins with the establishment of a health staff that is capable of providing CRD services effectively and compassionately.

## Priorities for Research and the Development of Research Capabilities

This review has uncovered a number of areas of ambiguity, which we have turned into research objectives for CRDs in LMICs (panel 2). These difficulties, however, cannot be solved without a robust critical mass of LMIC researchers. The American Thoracic Society/Pan African Thoracic Society's Methods course and the Structured Operational Research Training Initiative (SORT-IT) course, the Pan African Thoracic Society Methods in Epidemiologic, Clinical and Operations Research (PATS-MECOR) course in epidemiological, clinical, and operational research is an example of a successful respiratory-focused program that provides training and networking opportunities for research-interested individuals, clinicians from LMICs are needed to help enhance this competence. SORT-IT and PATS-MECOR both concentrate on clinical, epidemiological, and operational research, or the “science of doing better” (134, 135). Concept formulation, grant and protocol writing, quality-assured data gathering and analysis, and paper writing are all covered in detail in each session. Participants must meet numerous goals in order to advance, and substantial, hands-on mentoring is provided throughout. Over 1,000 participants from 90 countries contributed to a huge amount of published research that has influenced policy and practice in LMICs (134–139). Graduates have a proven track record of success in the workplace. Graduates have a great track record of staying in research after completing their courses (140–143) or could pursue a career as a course instructor (140–144).

## Conclusion

Chronic respiratory diseases have a significant role in the burden of illness in LMICs. Achieving the SDGs will necessitate taking steps to reduce illness burdens *via* better prevention and treatment. Poverty reduction initiatives must be at the forefront of preventative efforts, with a particular focus on maternal nutrition and health, lowering airborne pollutants (tobacco smoke, home and atmospheric air pollution, and occupational exposures), and improving the prevention and management of severe or untreated respiratory diseases, such as TB, especially in children and adolescents. Policy actions aimed at addressing these causes of CRDs will produce both short-term and long-term advantages. However, a significant burden of illness is expected to persist, necessitating evidence-based therapy options to minimize continuing disease and death in persons with established CRDs. In LMICs, better data on the epidemiology of CRDs and associated risk factors are required. Many information gaps still exist, and extrapolating data from HICs risks ignoring the particular exposures, health system limits, and social and political factors that define illnesses in LMICs. Understanding the etiology of CRDs and patient outcomes in LMICs and developing diagnostic and treatment techniques that are possible, acceptable, and suitable for local settings, will require renewed efforts. These techniques should take into account heterogeneity both within and across nations. In a world where people are migrating at an increasing rate, the applicability of results from LMICs to groups that have been forced or choose to migrate to other regions of the world should be explored as well (145). The universal health coverage agenda provides a perfect chance to guarantee that persons with CRDs who have affordable and long-term access to adequate and effective diagnostic assessment and pharmacological and non-pharmacological therapy interventions—goals that are applicable globally. CRD services will gain benefit from integration with wider tuberculosis and NCD care. The balance between programmatic methods aimed at delivering basic standardized interventions and customized methods aimed at targeting treatments more accurately requires careful study and should be adjusted to the local healthcare system. However, this will need resources and capacity building in all contexts, with special emphasis directed to the healthcare system's most remote levels. This objective will be difficult to achieve for many LMICs, but it emphasizes the need of improving health systems, capacity building, and implementation research in realizing the potential of universal health coverage to lessen the global burden of CRDs.

## Author Contributions

MH, MS, NS, and SP: planning. NA, MB, and QJ: data compilation. L-HZ, MoF, AK, MeF, SS, AA, and SKS: writing. L-HZ, TF, AA, IK, TF, and XW: proof reading. All authors contributed to the article and approved the submitted version.

## Funding

This work was supported by Nature Science Foundation of Zhejiang Province, China (No. LTY21H160001).

## Conflict of Interest

The authors declare that the research was conducted in the absence of any commercial or financial relationships that could be construed as a potential conflict of interest.

## Publisher's Note

All claims expressed in this article are solely those of the authors and do not necessarily represent those of their affiliated organizations, or those of the publisher, the editors and the reviewers. Any product that may be evaluated in this article, or claim that may be made by its manufacturer, is not guaranteed or endorsed by the publisher.

## References

[1] The World Bank. Low and Middle Income Countries. The World Bank. Available online at: https://data.worldbank.org/country/XO

[2] BennettJEStevensGAMathersCDBonitaRRehmJKrukME. NCD countdown 2030: worldwide trends in non-communicable disease mortality and progress towards sustainable development goal target 3.4. Lancet. (2018) 392:1072–88. 10.1016/S0140-6736(18)31992-530264707

[3] GlobalAgenda. Transforming our World: The 2030 Agenda for Sustainable Development. New York, NY: Division for Sustainable Development Goals (2015).

[4] EzzatiMPearson-StuttardJBennettJEMathersCD. Acting on non-communicable diseases in low-and middle-income tropical countries. Nature. (2018) 559:507–16. 10.1038/s41586-018-0306-930046068

[5] BukhmanGMocumbiAOAtunRBeckerAEBhuttaZBinagwahoA. The lancet NCDI poverty commission: bridging a gap in universal health coverage for the poorest billion. Lancet. (2020) 396:991–1044. 10.1016/S0140-6736(20)31907-332941823PMC7489932

[6] BushA. Lung development and aging. Am Thorac Soc. (2016) 13 (Suppl. 5):S438–46. 10.1513/AnnalsATS.201602-112AW28005431

[7] AgustíANoellGBrugadaJFanerR. Lung function in early adulthood and health in later life: a transgenerational cohort analysis. Lancet Respir Med. (2017) 5:935–45. 10.1016/S2213-2600(17)30434-429150410

[8] GrayDWillemseLVisagieACzövekDNduruPVankerA. Determinants of early-life lung function in African infants. Thorax. (2017) 72:445–50. 10.1136/thoraxjnl-2015-20740127856821PMC5520243

[9] AgrawalAAggarwalMSonnappaSBushA. Ethnicity and spirometric indices: hostage to tunnel vision? Lancet Respir Med. (2019) 7:743–4. 10.1016/S2213-2600(19)30204-831208952PMC6906084

[10] BurneyPHooperRJT. Forced vital capacity, airway obstruction and survival in a general population sample from the USA. Thorax. (2011) 66:49–54. 10.1136/thx.2010.14704120980245

[11] BurneyPJithooAKatoBJansonCManninoDNizankowska-MogilnickaE. Chronic obstructive pulmonary disease mortality and prevalence: the associations with smoking and poverty—a BOLD analysis. Thorax. (2014) 69:465–73. 10.1136/thoraxjnl-2013-20446024353008PMC3995258

[12] DuongMIslamSRangarajanSLeongDKurmiOTeoK. Mortality and cardiovascular and respiratory morbidity in individuals with impaired FEV1 (PURE): an international, community-based cohort study. Lancet Glob Health. (2019) 7:e613–23. 10.1016/S2214-109X(19)30070-131000131

[13] GrayDMTurkovicLWillemseLVisagieAVankerASteinDJ. Lung function in African infants in the drakenstein child health study. Impact of lower respiratory tract illness. Am J Respir Care Med. (2017) 195:212–20. 10.1164/rccm.201601-0188OC27509359PMC5394784

[14] LeeAGKaaliSQuinnADeliminiRBurkartKOpoku-MensahJ. Prenatal household air pollution is associated with impaired infant lung function with sex-specific effects. Evidence from graphs, a cluster randomized Cookstove intervention trial. Am J Respir Crit Care Med. (2019) 199:738–46. 10.1164/rccm.201804-0694OC30256656PMC6423100

[15] MacGintyRPKariukiSMBarnettWWedderburnCJHardyAHoffmanN. Associations of antenatal maternal psychological distress with infant birth and development outcomes: results from a South African birth cohort. Compr Psychiatry. (2020) 96:152128. 10.1016/j.comppsych.2019.15212831715335PMC6945113

[16] RanabhatCLJakovljevicMDhimalMKimCB. Structural factors responsible for universal health coverage in low-and middle-income countries: results from 118 countries. Front Public Health. (2020) 7:414. 10.3389/fpubh.2019.0041432039128PMC6985282

[17] FowlerMGQinMFiscusSACurrierJSFlynnPMChipatoT. Benefits and risks of antiretroviral therapy for perinatal HIV prevention. N Engl J Med. (2016) 375:1726–37. 10.1056/NEJMoa151169127806243PMC5214343

[18] BoltonCEBushAHurstJRKotechaSMcGarveyL. Lung consequences in adults born prematurely. Thorax. (2015) 70:574–80. 10.1136/thoraxjnl-2014-20659025825005

[19] HurstJRBeckmannJNiYBoltonCEMcEnieryCMCockcroftJR. Respiratory and cardiovascular outcomes in survivors of extremely preterm birth at 19 years. Am J Respir Crit Care Med. (2020) 202:422–32. 10.1164/rccm.202001-0016OC32302489PMC7397792

[20] VankerAGieRZarHJ. The association between environmental tobacco smoke exposure and childhood respiratory disease: a review. Expert Rev Respir Med. (2017) 11:661–73. 10.1080/17476348.2017.133894928580865PMC6176766

[21] FamorotiTSibandaWNdung'uTJB. Prevalence and seasonality of common viral respiratory pathogens, including cytomegalovirus in children, between 0–5 years of age in KwaZulu-Natal, an HIV endemic province in South Africa. BMC Pediatr. (2018) 18:240. 10.1186/s12887-018-1222-830031377PMC6054853

[22] SinaniotisCJ. Viral pneumoniae in children: incidence and aetiology. Paediatr Respir Rev. (2004) 5:S197–200. 10.1016/S1526-0542(04)90037-114980270

[23] LandriganPJSlyJLRuchirawatMSilvaERHuoXDiaz-BarrigaF. Health consequences of environmental exposures: changing global patterns of exposure and disease. Ann Glob Health. (2016) 82:10–9. 10.1016/j.aogh.2016.01.00527325064

[24] ZarHJBarnettWStadlerAGardner-LubbeSMyerLNicolMP. Aetiology of childhood pneumonia in a well vaccinated South African birth cohort: a nested case-control study of the drakenstein child health study. Lancet Respir Med. (2016) 4:463–72. 10.1016/S2213-2600(16)00096-527117547PMC4989125

[25] YoungSO'keeffePTArnottJLandauLI. Lung function, airway responsiveness, and respiratory symptoms before and after bronchiolitis. Arch Dis Child. (1995) 72:16–24. 10.1136/adc.72.1.167717730PMC1510966

[26] Organization WH. Global Tuberculosis Report 2019. Geneva: WHO (2018).

[27] MasekelaRAndersonRMoodleyTKitchinOPRisengaSMBeckerPJ. HIV-related bronchiectasis in children: an emerging spectre in high tuberculosis burden areas. Int J Tuberc Lung Dis. (2012) 16:114–9. 10.5588/ijtld.11.024422236856

[28] FerrandRADesaiSRHopkinsCElstonCMCopleySJNathooK. Chronic lung disease in adolescents with delayed diagnosis of vertically acquired HIV infection. Clin Infect Dis. (2012) 55:145–52. 10.1093/cid/cis27122474177PMC3369563

[29] GithinjiLNGrayDMHlengwaSMyerL. Lung function in South African adolescents infected perinatally with HIV and treated long-term with antiretroviral therapy. Ann Am Thorac Soc. (2017) 14:722–9. 10.1513/AnnalsATS.201612-1018OC28248548PMC5427744

[30] WoodruffAWEl SuniAKakuMAdamsonEAMaughanTSBundruN. Infants in Juba, southern Sudan: the first twelve months of life. Lancet. (1984) 324:506–9. 10.1016/S0140-6736(84)92577-76147559

[31] Ausloos M Local Local Burden of Disease Child Growth Failure Collaborators. Mapping child growth failure across low-and middle-income countries. J Nat. (2020) 577:231–4. 10.1038/s41586-019-1878-831915393PMC7015855

[32] BlackREVictoraCGWalkerSPBhuttaZAChristianPOnisDM. Maternal and child undernutrition and overweight in low-income and middle-income countries. Lancet. (2013) 382:427–51. 10.1016/S0140-6736(13)60937-X23746772

[33] FornoEWeinerDJMullenJSawickiGKurlandGHanYY. Obesity and airway dysanapsis in children with and without asthma. Am J Respir Crit Care Med. (2017) 195:314–23. 10.1164/rccm.201605-1039OC27552676PMC5328183

[34] HeinzerlingAPGuarnieriMJMannJKDiazJVThompsonLMDiazA. Lung function in woodsmoke-exposed guatemalan children following a chimney stove intervention. Thorax. (2016) 71:421–8. 10.1136/thoraxjnl-2015-20778326966237PMC10666195

[35] RylanceSNightingaleRNaunjeAMbalumeFJewellCBalmesJR. Lung health and exposure to air pollution in Malawian children (CAPS): a cross-sectional study. Thorax. (2019) 74:1070–7. 10.1136/thoraxjnl-2018-21294531467192PMC6860406

[36] GaudermanWJUrmanRAvolEBerhaneKMcConnellRRappaportE. Association of improved air quality with lung development in children. N Engl J Med. (2015) 372:905–13. 10.1056/NEJMoa141412325738666PMC4430551

[37] BalmesJR. How does diesel exhaust impact asthma? Thorax. (2011) 66:4–6. 10.1136/thx.2010.14539121149527

[38] BrunekreefBStewartAWAndersonHRLaiCKStrachanDP. Self-reported truck traffic on the street of residence and symptoms of asthma and allergic disease: a global relationship in ISAAC phase 3. Environ Health Perspect. (2009) 117:1791–8. 10.1289/ehp.080046720049134PMC2801184

[39] PandyaRJSolomonGKinnerABalmesJR. Diesel exhaust and asthma: hypotheses and molecular mechanisms of action. Environ Health Perspect. (2002) 110:103–12. 10.1289/ehp.02110s110311834468PMC1241152

[40] BarnesBR. Behavioural change, indoor air pollution and child respiratory health in developing countries: a review. Int J Environ Res Public Health. (2014) 11:4607–18. 10.3390/ijerph11050460724776723PMC4053881

[41] FaberTKumarAMackenbachJPMillettCBasuSSheikhA. Effect of tobacco control policies on perinatal and child health: a systematic review and meta-analysis. Lancet Public Health. (2017) 2:e420–37. 10.1016/S2468-2667(17)30144-528944313PMC5592249

[42] IfHM. Evaluation, Global Burden of Disease Collaborative Network. Global Burden of Disease Study 2016 (GBD 2016) Results. Institute for Health Metrics and Evaluation Seattle (2017).

[43] HalpinDMGCelliBRCrinerGJFrithPVarelaLSalviS. The GOLD summit on chronic obstructive pulmonary disease in low-and middle-income countries. Int J Tuberc Lung Dis. (2019) 23:1131–41. 10.5588/ijtld.19.039731718748

[44] CaballeroATorres-DuqueCAJaramilloCBolívarFSanabriaFOsorioP. Prevalence of COPD in five Colombian cities situated at low, medium, and high altitude (PREPOCOL study). Chest. (2008) 133:343–9. 10.1378/chest.07-136117951621

[45] EchazarretaALAriasSJDel OlmoRGiugnoERColodencoFDArceSC. Prevalence of COPD in 6 urban clusters in Argentina: the EPOC. AR study. Arch Bronconeumol. (2018) 54:260–9. 10.1016/j.arbr.2017.09.01729221827

[46] MenezesAMBPerez-PadillaRJardimJBMuiñoALopezMVValdiviaG. Chronic obstructive pulmonary disease in five Latin American cities (the PLATINO study): a prevalence study. Lancet. (2005) 366:1875–81. 10.1016/S0140-6736(05)67632-516310554

[47] BuistASMcBurnieMAVollmerWMGillespieSBurneyPManninoDM. International variation in the prevalence of COPD (the BOLD study): a population-based prevalence study. Lancet. (2007) 370:741–750. 10.1016/S0140-6736(07)61377-417765523

[48] MeghjiJNadeauGDavisKJWangDNyirendaMJGordonSB. Noncommunicable lung disease in sub-Saharan Africa. A community-based cross-sectional study of adults in urban Malawi. Am J Respir Crit Care Med. (2016) 194:67–76. 10.1164/rccm.201509-1807OC26788760PMC4960629

[49] ObasekiDOErhaborGEGnatiucLAdewoleOOBuistSA. Chronic airflow obstruction in a black African population: results of BOLD study, Ile-Ife, Nigeria. J Chron Obstruct Pulmon Dis. (2016) 13:42–9. 10.3109/15412555.2015.104110226451840

[50] WoldeamanuelGGMingudeAGetaB. Prevalence of chronic obstructive pulmonary disease (COPD) and its associated factors among adults in Abeshge District, Ethiopia: a cross sectional study. BMC Pulm Med. (2019) 19:181. 10.1186/s12890-019-0946-z31623601PMC6798340

[51] AgustíAFanerR. COPD beyond smoking: new paradigm, novel opportunities. Lancet Respir Med. (2018) 6:324–6. 10.1016/S2213-2600(18)30060-229496484

[52] SalviSSBarnesPJ. Chronic obstructive pulmonary disease in non-smokers. Lancet. (2009) 374:733–43. 10.1016/S0140-6736(09)61303-919716966

[53] Perez-PadillaRFernandezRVarelaMVLde OcaMMMuiñoATálamoC. Airflow obstruction in never smokers in five Latin American cities: the PLATINO study. Arch Med Res. (2012) 43:159–65. 10.1016/j.arcmed.2012.03.00722475778

[54] LamprechtBMcBurnieMAVollmerWMGudmundssonGWelteTNizankowska-MogilnickaE. COPD in never smokers: results from the population-based burden of obstructive lung disease study. Chest. (2011) 139:752–63. 10.1378/chest.10-125320884729PMC3168866

[55] LangePCelliBAgustíABoje JensenGDivoMFanerR. Lung-function trajectories leading to chronic obstructive pulmonary disease. N Engl J Med. (2015) 373:111–22. 10.1056/NEJMoa141153226154786

[56] TálamoCde OcaMMHalbertRPerez-PadillaRJardimJRBMuinoA. Diagnostic labeling of COPD in five Latin American cities. Chest. (2007) 131:60–7. 10.1378/chest.06-114917218557

[57] Casas HerreraAMontes de OcaMLópez VarelaMVAguirreCSchiaviEJardimJR. COPD underdiagnosis and misdiagnosis in a high-risk primary care population in four Latin American countries. A key to enhance disease diagnosis: the PUMA study. PLoS ONE. (2016) 11:e0152266. 10.1371/journal.pone.015226627073880PMC4830516

[58] LamprechtBSorianoJBStudnickaMKaiserBVanfleterenLEGnatiucL. Determinants of underdiagnosis of COPD in national and international surveys. Chest. (2015) 148:971–85. 10.1378/chest.14-253525950276

[59] VarelaMVLMuiñoAPadillaRPJardimJRTálamoCde OcaMM. Treatment of chronic obstructive pulmonary disease in 5 Latin American cities: the PLATINO study. Arch Bronconeumol. (2008) 44:58–64. 10.1016/S1579-2129(08)60016-618361870

[60] de OcaMMTálamoCPerez-PadillaRLopezMVMuiñoAJardimJRB. Use of respiratory medication in five Latin American cities: the PLATINO study. Pulm Pharmacol Ther. (2008) 21:788–93. 10.1016/j.pupt.2008.06.00318621136

[61] JardimJRStirbulovRMorenoDZabertGLopez-VarelaMV. Respiratory medication use in primary care among COPD subjects in four Latin American countries. Int J Tuberc Lung Dis. (2017) 21:458–465. 10.5588/ijtld.16.063328284262

[62] VanjareNChhowalaSMadasSKodguleRGogtayJSalviS. Use of spirometry among chest physicians and primary care physicians in India. NPJ Prim Care Respir Med. (2016) 26:1–5. 10.1038/npjpcrm.2016.3627385406PMC4936052

[63] HalpinDMCelliBRCrinerGJFrithPVarelaMVLSalviS. It is time for the world to take COPD seriously: a statement from the GOLD board of directors. Eur Respir J. (2019) 54:1900914. 10.1183/13993003.00914-201931273036

[64] DivoMCoteCde TorresJPCasanovaCMarinJMPinto-PlataV. Comorbidities and risk of mortality in patients with chronic obstructive pulmonary disease. Am J Respir Crit Care Med. (2012) 186:155–61. 10.1164/rccm.201201-0034OC22561964

[65] SinghSJHalpinDMSalviSKirengaBJ. Exercise and pulmonary rehabilitation for people with chronic lung disease in LMICs: challenges and opportunities. Lancet Respir Med. (2019) 7:1002–4. 10.1016/S2213-2600(19)30364-931629670

[66] AsherIBissellKChiangCYEl SonyAEllwoodPGarcía-MarcosL. Calling time on asthma deaths in tropical regions—how much longer must people wait for essential medicines? Lancet Respir Med. (2019) 7:13–5. 10.1016/S2213-2600(18)30513-730553847

[67] BatemanEDHurdSSBarnesPJBousquetJDrazenJMFitzGeraldM. Global strategy for asthma management and prevention: GINA executive summary. Euro Respir J. (2008) 31:143–78. 10.1183/09031936.0013870718166595

[68] NetworkGA. The Global Asthma Report. Auckland: Global Asthma Network (2018).

[69] LenneyWBushAFitzgeraldDAFletcherMOstremAPedersenS. Improving the global diagnosis and management of asthma in children. Thorax. (2018) 73:662–9. 10.1136/thoraxjnl-2018-21162629870146

[70] KanXHChiangCYEnarsonDARaoHLChenQAït-KhaledN. Asthma as a hidden disease in rural China: opportunities and challenges of standard case management. Public Health Action. (2012) 2:87–91. 10.5588/pha.12.002526392959PMC4463046

[71] BritishThoracic Society Scottish Intercollegiate Guidelines Network. British guideline on the management of asthma. Thorax. (2008) 63:iv1–21. 10.1136/thx.2008.09774118463203

[72] ReddelHKFitzGeraldJMBatemanEDBacharierLBBeckerABrusselleG. GINA 2019: a fundamental change in asthma management: treatment of asthma with short-acting bronchodilators alone is no longer recommended for adults and adolescents. Euro Respir J. (2019) 53:1901046. 10.1183/13993003.01046-201931249014

[73] BatemanEDReddelHKO'ByrnePMBarnesPJZhongNKeenC. As-needed budesonide–formoterol versus maintenance budesonide in mild asthma. N Engl J Med. (2018) 378:1877–87. 10.1056/NEJMoa171527529768147

[74] BeasleyRHollidayMReddelHKBraithwaiteIEbmeierSHancoxRJ. Controlled trial of budesonide–formoterol as needed for mild asthma. N Engl J Med. (2019) 380:2020–30. 10.1056/NEJMoa190196331112386

[75] HardyJBaggottCFingletonJReddelHKHancoxRJHarwoodM. Budesonide-formoterol reliever therapy versus maintenance budesonide plus terbutaline reliever therapy in adults with mild to moderate asthma (PRACTICAL): a 52-week, open-label, multicentre, superiority, randomised controlled trial. Lancet. (2019) 394:919–28. 10.1016/S0140-6736(19)31948-831451207

[76] O'ByrnePMFitzGeraldJMBatemanEDBarnesPJZhongNKeenC. Inhaled combined budesonide–formoterol as needed in mild asthma. N Engl J Med. (2018) 378:1865–76. 10.1056/NEJMoa171527429768149

[77] SobierajDMWeedaERNguyenEColemanCIWhiteCMLazarusSC. Association of inhaled corticosteroids and long-acting β-agonists as controller and quick relief therapy with exacerbations and symptom control in persistent asthma: a systematic review and meta-analysis. JAMA. (2018) 319:1485–96. 10.1001/jama.2018.276929554195PMC5876810

[78] AdeGGninafonMTawoLAït-KhaledNEnarsonDA. Management of asthma in Benin: the challenge of loss to follow-up. Public Health Action. (2013) 3:76–80. 10.5588/pha.12.008026393001PMC4463093

[79] El SonyAIChiangCYMalikEHassanainSAHussienHKhamisAH. Standard case management of asthma in Sudan: a pilot project. Public Health Action. (2013) 3:247–52. 10.5588/pha.13.001926393039PMC4463127

[80] DharRSinghSTalwarDMohanMTripathiSKSwarnakarR. Bronchiectasis in India: results from the European multicentre bronchiectasis audit and research collaboration (EMBARC) and respiratory research network of India registry. Lancet Global Health. (2019) 7:e1269–79. 10.1016/S2214-109X(19)30327-431402007

[81] QuintJKMillettERJoshiMNavaratnamVThomasSLHurstJR. Changes in the incidence, prevalence and mortality of bronchiectasis in the UK from 2004 to 2013: a population-based cohort study. Euro Respir J. (2016) 47:186–93. 10.1183/13993003.01033-201526541539PMC4982534

[82] ChandrasekaranRMac AogáinMChalmersJDElbornSJ. Geographic variation in the aetiology, epidemiology and microbiology of bronchiectasis. BMC Pulm Med. (2018) 18:83. 10.1186/s12890-018-0638-029788932PMC5964678

[83] ShoemarkAOzerovitchLWilsonRJR. Aetiology in adult patients with bronchiectasis. Respir Med. (2007) 101:1163–70. 10.1016/j.rmed.2006.11.00817223027

[84] ChangABBrownNToombsMMarshRLReddingGJ. Lung disease in indigenous children. Paediatr Respir Rev. (2014) 15:325–32. 10.1016/j.prrv.2014.04.01624958089

[85] BoaventuraRSibilaOAgustiAChalmersJD. Treatable traits in bronchiectasis. Eur Respir J. (2018) 52:1801269. 10.1183/13993003.01269-201830190263

[86] MorrowBM. Airway clearance therapy in acute paediatric respiratory illness: a state-of-the-art review. South Afr J Physiother. (2019) 75:1295. 10.4102/sajp.v75i1.129531309166PMC6620562

[87] AllwoodBWMyerLBatemanED. A systematic review of the association between pulmonary tuberculosis and the development of chronic airflow obstruction in adults. Respiration. (2013) 86:76–85. 10.1159/00035091723652030

[88] ByrneALMaraisBJMitnickCDLeccaLMarksGB. Tuberculosis and chronic respiratory disease: a systematic review. Int J Infect Dis. (2015) 32:138–46. 10.1016/j.ijid.2014.12.01625809770

[89] AmaralAFCotonSKatoBTanWCStudnickaMJansonC. Tuberculosis associates with both airflow obstruction and low lung function: BOLD results. Euro Respir J. (2015) 46:1104–12. 10.1183/13993003.02325-201426113680PMC4594762

[90] MeghjiJSimpsonHSquireSBMortimerK. A systematic review of the prevalence and pattern of imaging defined post-TB lung disease. PLoS ONE. (2016) 11:e0161176. 10.1371/journal.pone.016117627518438PMC4982669

[91] MeghjiJLesoskyMJoekesEBandaPRylanceJGordonS. Patient outcomes associated with post-tuberculosis lung damage in Malawi: a prospective cohort study. Thorax. (2020) 75:269–78. 10.1136/thoraxjnl-2019-21380832102951PMC7063395

[92] KhosaCBhattNMassangoIAzamKSaathoffEBakuliA. Development of chronic lung impairment in Mozambican TB patients and associated risks. BMC Pulm Med. (2020) 20:127. 10.1186/s12890-020-1167-132381002PMC7203866

[93] MarxFMFloydSAylesHGodfrey-FaussettPBeyersN. High burden of prevalent tuberculosis among previously treated people in Southern Africa suggests potential for targeted control interventions. Euro Respir J. (2016) 48:1227–30. 10.1183/13993003.00716-201627390274PMC5512114

[94] BalasegaramMBrigdenG. Empiric tuberculosis treatment in retreatment patients in high HIV/tuberculosis-burden settings. Lancet Infect Dis. (2014) 14:795–6. 10.1016/S1473-3099(14)70881-325164192

[95] HoubenRMLalliMKranzerKMenziesNASchumacherSG. What if they don't have tuberculosis? The consequences and trade-offs involved in false-positive diagnoses of tuberculosis. Clin Infect Dis. (2019) 68:150–6. 10.1093/cid/ciy54429982375PMC6293007

[96] RomanowskiKBaumannBBashamCAKhanFAFoxGJ. Long-term all-cause mortality in people treated for tuberculosis: a systematic review and meta-analysis. Lancet Infect Dis. (2019) 19:1129–37. 10.1016/S1473-3099(19)30309-331324519

[97] DormanSESchumacherSGAllandDNabetaPArmstrongDTKingB. Xpert MTB/RIF Ultra for detection of *Mycobacterium tuberculosis* and rifampicin resistance: a prospective multicentre diagnostic accuracy study. Lancet Infect Dis. (2018) 18:76–84. 10.1016/S1473-3099(17)30691-629198911PMC6168783

[98] KendallEASchumacherSGDenkingerCMDowdyDW. Estimated clinical impact of the Xpert MTB/RIF ultra cartridge for diagnosis of pulmonary tuberculosis: a modeling study. PLoS Med. (2017) 14:e1002472. 10.1371/journal.pmed.100247229240766PMC5730108

[99] van KampenSCWannerAEdwardsMHarriesADKirengaBJChakayaJ. International research and guidelines on post-tuberculosis chronic lung disorders: a systematic scoping review. BMJ Glob Health. (2018) 3:e000745. 10.1136/thorax-2018-212555.37930057796PMC6058174

[100] AllwoodBWVan Der ZalmMMAmaralAFSByrneADattaSEgereU. Post-tuberculosis lung health: perspectives from the first international symposium. Int J Tuberc Lung Dis. (2020) 24:820–828. 10.5588/ijtld.20.006732912387

[101] DlodloRABrigdenGHeldalEAllwoodBChiangCYFujiwaraPI. Management of Tuberculosis: a Guide to Essential Practice. Paris: International Union Against Tuberculosis and Lung Disease (2020).

[102] AndréjakCNielsenRThomsenVØDuhautPSørensenHT. Chronic respiratory disease, inhaled corticosteroids and risk of non-tuberculous mycobacteriosis. Thorax. (2013) 68:256–62. 10.1136/thoraxjnl-2012-20177222781123

[103] DongYHChangCHWuFLLShenLJCalverleyPMLöfdahlCG. Use of inhaled corticosteroids in patients with COPD and the risk of TB and influenza: a systematic review and meta-analysis of randomized controlled trials. Chest. (2014) 145:1286–97. 10.1378/chest.13-213724504044

[104] LeeCHKimKHyunMKJangEJLeeNRYimJJ. Use of inhaled corticosteroids and the risk of tuberculosis. Thorax. (2013) 68:1105–13. 10.1136/thoraxjnl-2012-20317523749841

[105] JonesRKirengaBJKatagiraWSinghSJPoolerJOkweraA. A pre–post intervention study of pulmonary rehabilitation for adults with post-tuberculosis lung disease in Uganda. Int J Chron Obstruct Pulmon Dis. (2017) 12:3533. 10.2147/COPD.S14665929270007PMC5729823

[106] HarriesADDlodloRABrigdenGMortimerKJensenPFujiwaraPI. Should we consider a ‘fourth 90'for tuberculosis?. Int J Tuberc Lung Dis. (2019) 23:1253–6. 10.5588/ijtld.19.047131753065

[107] RanzaniOTRodriguesLCBombardaSMintoCMWaldmanEA. Long-term survival and cause-specific mortality of patients newly diagnosed with tuberculosis in São Paulo state, Brazil, 2010–15: a population-based, longitudinal study. Lancet Infect Dis. (2020) 20:123–32. 10.1016/S1473-3099(19)30518-331676242PMC6928568

[108] World Health Organization. Monitoring the Building Blocks of Health Systems: A Handbook of Indicators and Their Measurement Strategies. Tanzania: World Health Organization (2010). Available online at: https://www.who.int/healthinfo/systems/WHO_MBHSS_2010_full_web.pdf

[109] BuistASParryV. The American thoracic society methods in epidemiologic, clinical, and operations research program. A research capacity-building program in low-and middle-income countries. Ann Am Thorac Soc. (2013) 10:281–9. 10.1513/Annals,AT.S.201304-081O.T23952845

[110] WHO. Assessing, National Capacity for the Prevention and Control of Noncommunicable Diseases. WHO (2012).

[111] World Health Organization. Noncommunicable Diseases Country Profiles. WHO (2018).

[112] TroegerCEKhalilIABlackerBFBiehlMHAlbertsonSBZimsenSR. Quantifying risks and interventions that have affected the burden of lower respiratory infections among children younger than 5 years: an analysis for the global burden of disease study 2017. Lancet Infect Dis. (2020) 20:60–79. 10.1016/S1473-3099(19)30410-431678026PMC7185492

[113] Vazquez-GarciaJCSalas-HernandezJPadillaRPde OcaM. M. Respiratory health in Latin America: number of specialists and human resources training. Arch Bronconeumol. (2014) 50:34–9. 10.1016/j.arbr.2013.12.00324119687

[114] ObasekiDAdeniyiBKolawoleTOnyedumCErhaborG. Gaps in capacity for respiratory care in developing countries. Nigeria as a case study. Ann Am Thorac Soc. (2015) 12:591–8. 10.1513/AnnalsATS.201410-443AR25734613

[115] ZarHJVankerAGrayDZampoliM. The African pediatric fellowship training program in pediatric pulmonology: a model for growing African capacity in child lung health. Ann Am Thorac Soc. (2017) 14:500–4. 10.1513/AnnalsATS.201612-953PS28125277

[116] WilmshurstJMMorrowBdu PreezAGithangaDKennedyN. The African pediatric fellowship program: training in Africa for Africans. Pediatrics. (2016) 137:1–12. 10.1542/peds.2015-274126659458

[117] MashBFairallLAdejayanOIkpefanOKumariJMatheeS. A morbidity survey of South African primary care. PLoS ONE. (2012) 7:e32358. 10.1371/annotation/3545077e-aded-4eef-a460-be1edbd1845c22442666PMC3306367

[118] CornickRPickenSWattrusCAwotiwonACarkeekEHanningtonJ. The practical approach to care kit (PACK) guide: developing a clinical decision support tool to simplify, standardise and strengthen primary healthcare delivery. BMJ Glob Health. (2018) 3:e000962. 10.1136/bmjgh-2018-00096230364419PMC6195147

[119] FairallLCornickRBatemanE. Empowering frontline providers to deliver universal primary healthcare using the practical approach to care kit. BMJ. (2018) 363:k4451. 10.1136/bmj.k445130355721PMC6200083

[120] World Health Organization. Implementation Tools: Package of Essential Noncommunicable (PEN) Disease Interventions for Primary Health Care in Low-Resource Settings. WHO (2013).

[121] World Health Organization. IMAI District Clinician Manual: Hospital Care Adolescents and Adults: Guidelines for the Management of Illnessess With Limited-Resources. WHO (2012).

[122] Fairall PL,. The Knowledge Translation Unit, University of Cape Town. Practical Approach to Care Kit (PACK): PACK Overview. (2020). Available online at: https://knowledgetranslation.co.za/pack/

[123] PickenSHanningtonJFairallLDohertyTBatemanERichardsM. PACK child: the development of a practical guide to extend the scope of integrated primary care for children and young adolescents. BMJ Glob Health. (2018) 3:e000957. 10.1136/bmjgh-2018-00095730397519PMC6203049

[124] CornickRWattrusCEastmanTRasCJAwotiwonAAndersonL. Crossing borders: the PACK experience of spreading a complex health system intervention across low-income and middle-income countries. BMJ Glob Health. (2018) 3(Suppl. 5):e001088. 10.1136/bmjgh-2018-00108830483416PMC6231097

[125] WattrusCZepedaJCornickRVZontaRde AndradeMPFairallL. Using a mentorship model to localise the practical approach to care kit (PACK): from South Africa to Brazil. BMJ Glob Health. (2018) 3(Suppl 5):e001016. 10.1136/bmjgh-2018-00101630483415PMC6231100

[126] AwotiwonASwordCEastmanTRasCJAnaPCornickRV. Using a mentorship model to localise the practical approach to care kit (PACK): from South Africa to Nigeria. BMJ Glob Health. (2018) 3:e001079. 10.1136/bmjgh-2018-00107930397520PMC6202991

[127] ZwarensteinMFairallLRLombardCMayersPBheekieAEnglishRG. Outreach education for integration of HIV/AIDS care, antiretroviral treatment, and tuberculosis care in primary care clinics in South Africa: PALSA PLUS pragmatic cluster randomised trial. BMJ. (2011) 342:d2022. 10.1136/bmj.d202221511783PMC3080737

[128] FairallLBachmannMOZwarensteinMBatemanEDNiessenLWLombardC. Cost-effectiveness of educational outreach to primary care nurses to increase tuberculosis case detection and improve respiratory care: economic evaluation alongside a randomised trial. Trop Med Int Health. (2010) 15:277–86. 10.1111/j.1365-3156.2009.02455.x20070633

[129] FairallLRFolbNTimmermanVLombardCSteynKBachmannMO. Educational outreach with an integrated clinical tool for nurse-led non-communicable chronic disease management in primary care in South Africa: a pragmatic cluster randomised controlled trial. PLoS Med. (2016) 13:e1002178. 10.1371/journal.pmed.100217827875542PMC5119726

[130] HannonBZimmermannCKnaulFMPowellRAMwangi-PowellFN. Provision of palliative care in low-and middle-income countries: overcoming obstacles for effective treatment delivery. J Clin Oncol. (2016) 34:62–8. 10.1200/JCO.2015.62.161526578612

[131] MasekelaRHallGLStanojevicSSartoriusBMacGintyRSaadHB. An urgent need for african spirometry reference equations: the paediatric and adult African Spirometry study. Int J Tuberc Lung Dis. (2019) 23:952–8. 10.5588/ijtld.18.044231533886

[132] FonjungoPNKebedeYMesseleTAyanaGTibessoGAbebeA. Laboratory equipment maintenance: a critical bottleneck for strengthening health systems in sub-Saharan Africa?. J Public Health Policy. (2012) 33:34–45. 10.1057/jphp.2011.5722071568

[133] AgodokpessiGAït-KhaledNGninafonMTawoLBekouWPerrinC. Assessment of a revolving drug fund for essential asthma medicines in Benin. J Pharm Policy Pract. (2015) 8:1–8. 10.1186/s40545-015-0033-725914829PMC4394562

[134] ZachariahRHarriesADIshikawaNRiederHLBissellKLasersonK. Operational research in low-income countries: what, why, and how?. Lancet Infect Dis. (2009) 9:711–7. 10.1016/S1473-3099(09)70229-419850229

[135] RamsayAHarriesADZachariahRBissellKHinderakerSGEdgintonM. The structured operational research and training initiative for public health programmes. Public Health Action. (2014) 4:79–84. 10.5588/pha.14.001126399203PMC4539036

[136] TripathyJPKumarAMGuillermNBergerSDBissellKReidA. Does the structured operational research and training initiative (SORT IT) continue to influence health policy and/or practice?. Glob Health Action. (2018) 11:1500762. 10.1080/16549716.2018.150076230080987PMC6084496

[137] KumarAMZachariahRSatyanarayanaSReidAJVan den BerghRTayler-SmithK. Operational research capacity building using ‘the union/MSF'model: adapting as we go along. BMC Res Notes. (2014) 7:819. 10.1186/1756-0500-7-81925409542PMC4253003

[138] SagiliKDSatyanarayanaSChadhaSSWilsonNCKumarAMMoonanPK. Operational research within a global fund supported tuberculosis project in India: why, how and its contribution towards change in policy and practice. Glob Health Action. (2018) 11:1445467. 10.1080/16549716.2018.144546729553308PMC5912428

[139] ZachariahRGuillermNBergerSKumarAMSatyanarayanaSBissellK. Research to policy and practice change: is capacity building in operational research delivering the goods? Trop Med Int Health. (2014) 19:1068–75. 10.1111/tmi.1234324909292

[140] GuillermNBissellKKumarAMVRamsayAReidAJZachariahR. Sustained research capacity after completing a structured operational research and training (SORT IT) course. Public Health Action. (2016) 6:207–8. 10.5588/pha.16.005727695687PMC5034790

[141] GuillermNTayler-SmithKBergerSDBissellKKumarAMVRamsayA. What happens after participants complete a Union-MSF structured operational research training course? Public Health Action. (2014) 4:89–95. 10.5588/pha.14.001426399205PMC4539032

[142] GuillermNTayler-SmithKDar BergerSBissellKKumarAMVRamsayA. Research output after participants complete a structured operational research and training (SORT IT) course. Public Health Action. (2015) 5:266–8. 10.5588/pha.15.004526767182PMC4682620

[143] BissellKHarriesADReidAJEdgintonMHinderakerSGSatyanarayanaS. Operational research training: the course and beyond. Public Health Action. (2012) 2:92–7. 10.5588/pha.12.002226392960PMC4463048

[144] FatimaRYaqoobAQadeerEHinderakerSGHeldalEZachariahR. Building sustainable operational research capacity in Pakistan: starting with tuberculosis and expanding to other public health problems. Glob Health Action. (2019) 12:1555215. 10.1080/16549716.2018.155521531154986PMC6327920

[145] Garcia-MarcosLRobertsonCFRoss AndersonHEllwoodPWilliamsHC. Does migration affect asthma, rhinoconjunctivitis and eczema prevalence? Global findings from the international study of asthma and allergies in childhood. Int J Epidemiol. (2014) 43:1846–54. 10.1093/ije/dyu14525056339

